The article "Physical Fitness Recovery of Athletes Based on High-Intensity Sports Intermittent Training" was retracted in 2023. Reasons: signs of a paper mill; compromised peer review; unreliable results or conclusions.

# Physical Fitness Recovery of Athletes Based on High-Intensity Sports Intermittent Training

**DOI:** 10.1155/2022/3370499

**Published:** 2022-07-26

**Authors:** Ruihua He, Xiwen Yang, Ligang Ma

**Affiliations:** ^1^Capital University of Physical Education and Sports, Beijing, 100191, China; ^2^Pingxiang University, Pingxiang, 337055, Jiangxi, China; ^3^Hebei University of Engineering, Handan, 056038, Hebei, China

## Abstract

Baseball itself is a new sport. In the process of training, teachers often use traditional training methods, which leads to unsatisfactory training results. High-intensity intermittent and intensive interval training can better improve the efficiency of athletes' oxidation and energy supply and ultimately play a positive role in improving athletes' performance. This paper takes the influence of high-intensity and intensive interval training on the special endurance of baseball players as the research object. A series of functional training programs are developed through adaptive training, testing, coordination training, and recovery training. Through the use of experimental means to understand the influence of high-intensity interval training and intensive interval training on the physical fitness of baseball players, the paper is aimed at providing ways and means to improve the physical fitness level of baseball players in the future. Based on the experimental test data, functional training is different from traditional training methods to make up for the lack of training research. It is to improve the competitive ability of our baseball players and promote the development of our baseball. It plays an active role in improving the specific endurance, speed, and intermittent endurance of baseball players.

## 1. Introduction

Baseball is a more intense sport, which requires athletes to touch or fight with their bodies, so the rate of physical contact is very high. To achieve good training results, athletes themselves need to train in endurance, speed, and coordination ability. At the same time, baseball has the characteristics of total defense and total attack. There are high requirements for athletes' running ability, speed, and endurance. There is no linear and stable standard for running and running speed in competition [1]. Special speed, endurance, and physical strength can enable athletes to adapt to various requirements of different competition environments. In baseball, athletes must run fast in different distances and directions and need enough physical strength to cope with the game. The strength of special endurance quality directly affects the normal play of athletes' techniques and tactics [2].

The principle of interval training is to “pay attention to the basic posture of the body and the mode of human movement, integrate the various qualities of the body to optimize the most basic sports ability of the human body, and systematically optimize the mode of movement, spinal strength, power chain, recovery, and regeneration.” At the same time, with the continuous advancement of technology, interval training has been optimizing and enriching itself for different training objects and training contents [3]. With the maturity of the FMS (functional movement screen) evaluation system and wide recognition in the industry, it has passed interval training testing methods such as FMS and YBT. It makes up for the shortcomings of traditional training tests for many sports training research and evaluation systems and proves the scientificity and authority of the interval training [4].

In recent years, the breadth and depth of research on “interval training” have been gradually accelerated, which proves the value of “interval training” for different groups of people and the potential that can be developed. In the study of training methods for any project, interval training still has great attraction and depth of study [5].

Tabata believes that functional training has a wide range of significance. Functional training can not only adapt to and conform to the training characteristics of various sports but also make adaptive adjustments according to the training content. All training is based on the purpose of actual combat and is summed up in functional training [6]. He believes the following: first, the ability of coordination in sports is the basis of left and right training; training movements is not to train muscles but to train movement skills, and then, train special sports skills. Second, first develop the core strength and then develop the body strength; first use the self-weight training and then use resistance training. Third, first train strength and then train strength endurance; first train speed and then train speed endurance. Using the unique adaptability of the human body can enhance the integrity of the movement structure without physical changes. People can enhance the control and integrity of their movement by increasing muscles. Each link can be achieved through the coordination of the various links of the human body. At the same time, it can also improve sports skills and reduce unnecessary sports injuries, improve the control of the brain and nerves over the body, and reflect the characteristics of functional training [7].

Martijn et al. created the theory of the “IHP” functional training method, which divides human body movement into four categories: push and pull, rotation, horizontal movement, and vertical movement, and it was called “four pillars movement” [8]. Also known as the functional principle of “IHP” training, Alan et al. believe that “functional training is to integrate the overall target movements with certain sports mechanics characteristics and requirements into the training” [9].

Henderson et al. believe that functional training is holistic training involving multiple muscle groups and joints in actual sports, rather than a single local limb activity [10]. Through functional training mode, athletes' body movements can reach the required level of economy, stability, and efficiency. At the same time, it can also ensure the improvement of human sports ability and prevent sports injuries [11].

At present, interval training is still a new field of training and research in China and abroad, but its interval training is mainly manifested in low space requirements, low equipment requirements, and high time freedom. The training method is flexible and changeable, which can carry out interval training for athletes of different events and at the same training stage and can combine multidimensional training methods to carry out efficient sports training to achieve training results. It makes the training of interval training in various projects more frequent and in-depth and also more in-depth and feasible [12].

Combined with the characteristics of baseball, the high-intensity interval and intensive interval training designed in this paper adhere to certain principles to ensure the reliability and practicability of training methods and save the training time of athletes. High-intensity interval training and intensive interval training have some differences in specific training arrangements and high-intensity interval training. The training load time is controlled below 40 seconds. The heart rate of baseball players is always monitored during the training process, and the heart rate in the training state is controlled at 190 times per minute. The essence of high-intensity interval training is to train with a heavy load in a short interval to promote the physical fitness of baseball players. After high-intensity interval training, the special endurance of athletes in the intermittent training group has been greatly improved. The anaerobic endurance quality has been improved faster, and the performance of athletes has been significantly improved.

## 2. Related Work

### 2.1. High-Intensity Interval Training

The English name of high-intensity interval training is also called HIIT, which means that the intensity of its load will be greater than the anaerobic threshold. Its duration is 10 seconds to 5 minutes in the middle of the short track. The intensity of its interval belongs to the exercise content of low intensity and resting intensity. Compared with the traditional means, the advantages of this training method are more obvious, and it has the characteristics of high competitiveness and practicability [13].

### 2.2. Intensive Interval Training

Intensive interval training is one of the means of exercise training. It is an aerobic training method. It plays an active role in training aerobic metabolism, glycolysis, and cardiopulmonary function. Training by this means can be very important for related sports such as speed endurance and strength endurance, which are dominated by physical fitness [14]. In the process of using this training method, the essential difference between intensive interval training and high-intensity interval training is that the interval time of training in the training unit is different. The interval time of intensive interval training is between 100 and 300 seconds, and the training intensity is controlled between 5% and 10% of the intensity of sports events [15].

## 3. Enhanced Interval Training Program

The intensive interval training protocol is shown in Table 1. The interval training group was given high-intensity interval training, while the traditional training group was given intensive interval training.

## 4. Consultation of Expert Opinions

The first round of expert investigation was carried out according to the initially designed questionnaire. In the first round of investigation, experts were invited to score the importance of the general physical fitness index and specific physical ability index of baseball designed in the questionnaire. The evaluation of the importance of general physical fitness indicators and specific physical ability indicators in baseball is divided into five dimensions: very important, relatively important, general, relatively unimportant, and very unimportant. The score of each dimension is 5 points, 4 points, 3 points, 2 points, and 1 point. Experts score according to the importance of the indicators. Finally, the results of the general physical fitness index and specific physical ability index of baseball are formed [16]. The preliminary expert opinion form is shown in Table 2.

The average score and standard deviation are selected as the basis for the importance of the indicator. The average score of the indicator is the average value of the importance score of each expert in the indicator, and the score range is between 1 and 5. The higher the average score is, the higher the importance of the indicator is. The standard deviation is the degree of deviation of the score of each expert in the importance score [17].

## 5. Reliability Index Analysis

To ensure the reliability of the study, three indicators including coefficient of variation, Kendall concordance coefficient (Kendall), and chi-square test were selected for reliability analysis [18].

1. The coefficient of variation is an index reflecting the degree of dispersion of probability distribution. The basic condition used is that the average value is not zero. In the process of consulting the general physical fitness index and specific physical ability index of baseball, the coefficient of variation is used to evaluate the degree of dispersion of expert scoring results [19]. The calculation formula of the coefficient of variation is

(1) $$\begin{array}{c} \text{CV}=\frac{\text{Standard Deviation}}{\text{The average value}}\times 100\%, \end{array}$$

where CV is the coefficient of variation. The smaller the CV calculation result is, the more consistent the experts' scoring opinions are.

(2) Kendall concordance coefficient (KendallW) is a relevant quantity to measure the difference of SPSS nonparametric test, which can be used as an index to test the consistency of expert opinions. The calculation result of Kendall concordance coefficient is between 0 and 1. The larger the calculation result of Kendall concordant coefficient is, the higher the degree of coordination between values is. This means that the degree of agreement among experts is higher [20]. The formula is

(2) $$\begin{array}{c} w=\sqrt{\frac{s}{k^{2}\left(N^{3}-N\right)-k\sum_{i=1}^{k}T_{i}}}, \end{array}$$

where *w* represents Kendall's concordance coefficient, *N* represents the number of indicators, *K* represents the number of experts, and *T* represents the square difference of the sum of the importance scores of each indicator.

(3) The chi-square test is a method to test the distribution of numerical values in a nonparametric test. The chi-square test can be used to evaluate the coordination degree of expert evaluation opinions. According to the final calculated *P* value, when *P* < 0.5, it shows that the coordination degree of expert evaluation results is higher, which reflects higher credibility under nonaccidental circumstances [21].

## 6. Experimental Results and Analysis

### 6.1. Experimental Protocol

The screening indicators such as 50 m, free bar bench press, standing long jump, repeated crossing, 3000 m, pull-up, finger push-up, and sitting forward bending were decomposed and expanded to determine the reselected indicators. The general physical fitness indicators were divided into four secondary indicators: 50 m, free bar bench press, standing long jump, and repeated crossing. The experts were consulted. The results are shown in Tables 3 and 4. Revise and optimize according to experts' suggestions, and finally determine the final index of the general physical fitness index [22].

The experts were consulted on the reselected indicators. In the first round, the scores were shown in Table 3. It can be seen that the scores of 50 m and standing long jump were more than 4 points. Therefore, the experts' suggestion for these two low-score training methods was to delete them, so it was suggested to delete them [23].

Based on the results of the first round of expert consultation, the second round of opinions is collected from the experts, and the results are shown in Table 4.

After the second round of expert consultation, the experts scored higher on the two indicators of 50 m and standing long jump. Thus, the two general physical fitness indicators of baseball players, namely, 50 m and standing long jump, were determined. The third round of questionnaire opinions was not collected [24].

### 6.2. Analysis of Experimental Results

#### 6.2.1. Comparison of Test Results of General Physical Fitness Indexes of Athletes in the Two Groups before and after the Experiment

The test results of general physical fitness indexes of athletes in the two groups before the experiment are shown in Table 5.

Before the experiment, the results of athletes' general physical fitness index test were basically the same.

1. The test results of the 50 m running (s) in the interval training group are shown in Table 6

The general physical fitness of athletes in the interval training group has been greatly improved, which shows that the high-intensity interval training can effectively improve the general physical fitness of male baseball players [25].

(2) The test results of 50 m running (s) in the traditional training group are shown in Table 7

Compared with the test results before the experiment, there was a significant difference. By using the same test comparison method, this paper tests the standing long jump performance of baseball players in the interval training group before and after the experiment. After five weeks of the experiment, the average performance of the players has increased by 3.75 cm, and the performance of the players has improved significantly. Ten weeks after the experiment, the average performance of players in the standing long jump is significantly different from that before the experiment. Under the intensive interval training method, the physical fitness of baseball players in the traditional training group has also been improved, and the improvement is also large, indicating that intensive interval training generally plays an active role in improving athletes.

#### 6.2.2. Comparison of Test Results of General Physical Fitness Indexes of Athletes in the Two Groups after the Experiment

1. The results of the general physical fitness index test in the interval training group at 5 weeks after the experiment are shown in Table 8

Five weeks after the experiment, there is a certain gap between the average scores of athletes in the interval training group and the traditional training group in the 50-meter race. There was no significant difference in the baseball players in the interval training group. The speed and strength test results of baseball players in the interval training group were slightly better than those in the control group, but the overall difference was small, which indicates that the high-intensity interval and intensive interval training can quickly and effectively improve the speed quality of baseball players.

(2) The results of the general physical fitness index test in the interval training group at 10 weeks after the experiment are shown in Table 9

High-intensity interval training and intensive interval training are conducive to improving the general physical quality of baseball players. In contrast, high-intensity interval training is slightly better than intensive interval training in the training effect of explosive force quality.

(3) The experimental comparison test results are shown in Figure 1

In the high-intensity interval training and the intensive interval training, the athlete carries out the short-time and high-intensity training for a plurality of times and can carry out the training in a minimally mild exercise mode or a completely resting mode every two training times. In the process, a full-strength sprint mode is adopted, and the exercise time and the interval period can last for several seconds or several minutes each time. It effectively promotes the improvement of athletes' speed quality, strength quality, and explosive force.

#### 6.2.3. Analysis of the Influence of Specific Endurance Index

The screening indexes of 250 m sprint, 3000 m, 300 m turn-back run, YOYO test, 12 min run, wild horse run, 25 m Z-shaped run, and goal turn-back run were decomposed and expanded to determine the reselected indexes. The special endurance indexes were divided into five secondary indexes: 3000 m, YOYO test, 12 min run, wild horse run, and goal turn-back run. Consult the experts, modify and optimize according to the experts' suggestions, and finally determine the final index of the special endurance index.

The results of the first round of expert consultation on specific endurance indicators are shown in Table 10.

Based on the results of the first round of expert consultation, two rounds of opinions are collected from experts again, and the results are shown in Table 11.

After the second round of expert consultation, the scores of experts on the four indicators are higher than 4.7. The expert scoring results are higher, and the expert opinions are unified. All the four special quality indicators are retained, and the third round of expert consultation is no longer carried out.

#### 6.2.4. Comparison of Results of the Special Endurance Index Test

1. The results of the special endurance index test before the experiment are shown in Table 12

Before the experiment, there was no significant difference (*P* > 0.05) in the performance between the intermittent training group and the traditional training group, and the results of the special endurance index test were basically the same before the experiment.

(2) The test results of the specific endurance index of the interval training group are shown in Table 13

The results show that compared with before the experiment, the average performance of the athletes has increased by nearly 11 seconds. The average performance (*P* < 0.05) of the athletes has increased by nearly 23 seconds in the 10 weeks after the experiment. The performance has improved significantly, and there is a significant difference in the 10 weeks after the experiment. There was no significant difference (*P* > 0.05) between the athletes 5 weeks after the experiment and before the experiment. There was a significant difference between the average performance of athletes about the 300 m shuttle run 10 weeks after the experiment and before the experiment.

(3) The test results of the specific endurance index of the traditional training group are shown in Table 14

(4) The experimental comparison test results are shown in Figure 2

After 10 weeks of training, intensive interval training is faster and more effective in improving the aerobic endurance of baseball players, while longer training cycles are needed to improve the anaerobic endurance.

## 7. Conclusion

This paper takes the comparison of the effects of intensive interval training on the specific endurance of baseball players as the research object. In the interval training group, high-intensity interval training was used, while in the traditional training group, intensive interval training was used. The training time and intensity of the two groups were the same. Under the guidance of coaches, 8 weeks of high-intensity and intensive intervention training were carried out. In the course of the experiment, two groups of baseball players were tested before and after the experiment, and finally, the relevant data were obtained. In the process of data statistics, the SPSS25 software was used for statistical analysis. Two groups of special endurance changes before and after training were analyzed. The results were obtained, which effectively pointed out the effect of high-intensity interval and intensive interval training after the intervention. High-intensity interval training focuses on high-intensity and high-load training, which plays an active role in the development of baseball players' explosive power quality and anaerobic sports ability, but in the aspect of sustained endurance training, it needs a longer training cycle.

In future work, sports intelligent equipment should be applied to sports training and sports scientific research innovation. Whether athletes or coaches, they should take the initiative to change the lack of awareness in the training system and improve the baseball training system from the perspective of data.

## Figures and Tables

**Figure 1:** Experimental comparison test results (1).

**Figure 2:** Test results of specific endurance index (2).

**Table 1:** Formulation of training plan.

	Monday	Wednesday	Friday	Training monitoring
Interval training group	Carry out 40-second sprint with four times as a group and two large groups. The intensity is 40-second full sprint to exhaustion. The rest time ratio is 1 : 2, and the rest time between large groups is 10 minutes	Carry out a 30-second sprint with six times as a group and two large groups. The intensity is 30-second full sprint to exhaustion. The rest time ratio is 1 : 2, and the rest time between large groups is 10 minutes	Carry out 20-second sprint with four times as a group and three groups. The intensity is 20-second full sprint to exhaustion. The rest time ratio is 1 : 2, and the rest time between groups is 10 minutes	During each training, the intensity of exercise load is required to reach the corresponding heart rate standard, and the whole training process is required

Traditional training group	The 800 m interval training includes two trips as a large group and two large groups. The intensity of heart rate is 165-175 beats per minute. The rest time ratio is 1 : 4	The 600 m interval training includes 3 times as a group and 2 groups. The intensity of heart rate is 165-175 times/minute	The 250 m interval training includes 3 times as a group and 2 large groups. The intensity of heart rate is 175-185 times per minute, and the rest time ratio is 1 : 4.	Heart rate band monitoring

**Table 2:** Expert opinion request form (*N* = 10).

	Specific indicator
General physical indicator	50 m
	Liberal ring parallel
	Standing long jump
	Repeatedly cross

Special physical indicator	3000 m
	25mz running
	300 M back running
	Mustang run

**Table 3:** Results of the first round of expert consultation (*N* = 10).

Check the indicator	Average score	Standard deviation	Coefficient of variation	Kendall's coefficient of concordance	*P*
50 m	4.825	0.425	0.102	/	/
Free bar bench press	3.089	1.156	0.401	0.413	0.034
Standing long jump	4.521	0.398	0.104	/	/
Repeatedly across	3.482	0.392	0.098	/	/

**Table 4:** Results of the second round of expert consultation (*N* = 10).

Check the indicator	Average score	Standard deviation	Coefficient of variation	Kendall's coefficient of concordance	*P*
50 m	4.814	0.157	0.033	0.516	0.001
Standing long jump	4.742	0.324	0.047	/	/

**Table 5:** Test results of athletes' general physical fitness indexes before the experiment.

	50-meter running (s)	Standing long jump (cm)
Interval training group	6.82 ± 0.31	282.37 ± 7.512
Traditional training group	6.94 ± 0.32	24.71 ± 8.77
*P*	0.781	0.887

**Table 6:** Test results of general physical fitness indexes in the interval training group.

	Scores		*P*
50 meters running (s)	Before the experiment	6.87 ± 0.32	/
	5 weeks after the experiment	6.55 ± 0.34	0.015
	10 weeks after the experiment	6.42 ± 0.31	0.001

Standing long jump (cm)	Before the experiment	278.69 ± 8.21	/
	5 weeks after the experiment	282.44 ± 9.34	0.042
	10 weeks after the experiment	285.67 ± 7.41	0.004

**Table 7:** Test results of general physical fitness indexes of the traditional training group.

	Scores		*P*
50-meter running (s)	Before the experiment	6.91 ± 0.31	/
	5 weeks after the experiment	6.66 ± 0.33	0.03
	10 weeks after the experiment	6.44 ± 0.38	0.001

Standing long jump (cm)	Before the experiment	277.44 ± 9.14	/
	5 weeks after the experiment	281.35 ± 8.67	0.057
	10 weeks after the experiment	285.14 ± 7.76	0.015

**Table 8:** Test results of general physical fitness indexes 5 weeks after the experiment.

	50-meter running (s)	Standing long jump (cm)
Interval training group	6.55 ± 0.34	282.44 ± 9.34
Traditional training group	6.66 ± 0.33	281.35 ± 8.67
*P*	0.653	0.859

**Table 9:** Test results of general physical fitness indexes 10 weeks after the experiment.

	50-meter running (s)	Standing long jump (cm)
Interval training group	6.42 ± 0.31	285.67 ± 7.41
Traditional training group	6.44 ± 0.38	285.14 ± 7.76
*P*	0.908	0.913

**Table 10:** The results of the first round of expert consultation on specific endurance indicators (*N* = 10).

Check the indicators	Average scores	Standard deviation	Coefficient of variation	Kendall's coefficient of concordance	*P*
3000 m	4.661	0.647	0.139	/	/
25 m Z-run test	3.467	0.812	0.234	/	/
250 m sprint	4.689	0.671	0.143	0.356	
Wild horse run	3.343	1.321	0.395	/	/
300 m back and forth run	4.847	1.671	0.345	/	

**Table 11:** Results of the second round of expert consultation on general physical fitness indicators (*N* = 10).

Check the indicators	Average scores	Standard deviation	Coefficient of variation	Kendall's coefficient of concordance	*P*
3000 m	4.784	0.211	0.044	/	/
300 m back and forth run	4.802	0.109	0.023	0.337	0.011
250 m sprint	4.775	0.214	0.045	/	
YOYO running	4.703	0.238	0.051	/	/

**Table 12:** Test results of athletes' special endurance indexes before the experiment.

	3000 m running (s)	300 m back and forth run (s)
Interval training group	767.45 ± 42.34	57.88 ± 4.59
Traditional training group	762.57 ± 49.41	58.92 ± 4.43
*P*	0.903	0.745

**Table 13:** Test results of specific endurance indexes of athletes in the interval training group before and after the experiment.

Test indicators	Stage	Scores	*P*
3000 m (s)	Before experiment	767.45 ± 42.34	/
	Five weeks after the experiment	756.57 ± 49.54	0.057
	Ten weeks after the experiment	744.77 ± 40.47	0.032

300 m back and forth run (s)	Before experiment	57.88 ± 4.59	/
	Five weeks after the experiment	55.81 ± 5.54	0.034
	Ten weeks after the experiment	54.19 ± 6.17	0.015

**Table 14:** Test results of special endurance indexes of athletes in the traditional training group before and after the experiment.

Test indicators	Stages	Scores	*P*
3000 m (s)	Before experiment	762.57 ± 49.41	/
	Five weeks after the experiment	754.01 ± 41.24	0.045
	Ten weeks after the experiment	742.47 ± 49.81	0.006

300 m back and forth run (s)	Before experiment	58.92 ± 4.43	/
	Five weeks after the experiment	58.55 ± 5.51	0.713
	Ten weeks after the experiment	56.04 ± 4.17	0.048

## Data Availability

The data used to support the findings of this study are available from the corresponding author upon request.
